# CUL4B promotes aggressive phenotypes of HNSCC via the activation of the Wnt/β‐catenin signaling pathway

**DOI:** 10.1002/cam4.1960

**Published:** 2019-03-18

**Authors:** Yuanyuan Wang, Dan Yue

**Affiliations:** ^1^ Department of Anesthesiology, The Fourth Affiliated Hospital China Medical University Shenyang China; ^2^ Department of Laboratory Medicine ShengJing Hospital of China Medical University Shenyang China

**Keywords:** angiogenesis, CUL4B, HNSCC, metastasis, Wnt/β‐catenin signaling

## Abstract

Previous studies have revealed that CUL4B is overexpressed in various types of cancer and that its overexpression is related to the progression and metastasis of tumors. However, the biological functions of CUL4B in the progression of head and neck squamous cell carcinoma (HNSCC) are still not well understood. In the current study, we aimed to determine the changes in biological functions and molecular events that are related to CUL4B overexpression. Interestingly, our results showed that CUL4B is upregulated in HNSCC and that its upregulation is associated with poor survival and worse histological grade. Overexpression of CUL4B promoted cancer cell growth, invasion, and migration, as well as epithelial‐mesenchymal transition, whereas the loss of CUL4B abrogated these malignant phenotypes. Moreover, our mechanistic investigations suggest that the Wnt/β‐catenin signaling pathway was activated by CUL4B overexpression. Treatment with a Wnt/β‐catenin inhibitor decreased CUL4B‐induced migration and invasion, establishing a key role of Wnt/β‐catenin signaling in mediating the effects of CUL4B expression. Together, these results demonstrate a key contribution of CUL4B overexpression in the malignant behavior of HNSCC cells, at least in part through the stimulation of angiogenesis and the activation of the Wnt/β‐catenin signaling pathway.

## 1 INTRODUCTION

Head and neck squamous cell carcinoma (HNSCC) accounts for approximately six percent of all cancers; it is the sixth most common cancer in the world.^1^ There are approximately 650 000 new HNSCC cases and 350 000 HNSCC‐related deaths each year.^2^ Although there has been considerable progress made in the diagnosis and treatment of HNSCC, the prognosis of HNSCC patients is still unsatisfactory.^3^ Conventional therapy for HNSCC has limited efficacy and substantial side effects due to the lack of specificity.^4^ However, recent progress in the treatment of HNSCC and the study of the underlying molecular mechanisms have produced a slight increase in the 5‐year survival rate, although it is still close to 50%.^5^ In addition, various biomarkers have been shown to be associated with the progression of HNSCC.^6^, ^7^ The identification and verification of prognostic factors can improve treatment as a complement to clinical histopathology.

Cullin 4B (CUL4B), a scaffold protein that assembles CRL4B ubiquitin ligase complexes, is overexpressed in a number of solid malignancies, and it silences tumor suppressors in a post‐transcriptional manner.^8^, ^9^ Previous studies have revealed that CUL4B expression is enhanced in breast cancer cells and human hepatocellular carcinoma, and its overexpression predicts poor prognosis and promotes tumor cell proliferation.^10^, ^11^ It has been demonstrated that CUL4B together with Myc can promote tumor cell proliferation.^12^ However, it is not well understood whether CUL4B exerts any of these effects in the development of human HNSCC. This prompted us to investigate the role of CUL4B in HNSCC.

The Wnt/β‐catenin signaling pathway is conserved throughout evolution and is crucial during both normal embryonic development and throughout the life to maintain homeostasis of in virtually every tissue. The Wnt/β‐catenin pathway is initiated by Wnt family ligands, secreted lipoglycoproteins that act to the frizzled (FZD) family receptors. The accumulated nuclear β‐catenin can interact directly with T‐cell transcription factor (TCF) and other factors to drive specific gene expression, potentially activating genes involved in proliferation and transformation.

Our results indicated that CUL4B promotes HNSCC cell growth and metastasis via stimulating angiogenesis and activating the Wnt/β‐catenin signaling pathway. These results suggest that the level CUL4B is a marker of therapeutic efficacy and a promising target in the treatment of HNSCC.

## 2 MATERIALS AND METHODS

### 2.1 Cell culture and reagents

The human HNSCC cell line JHU‐012 was procured from American Type Culture Collection (Manassas, VA, USA) and cultured in RPMI‐1640 medium supplemented with 100 µg/mL streptomycin, 100 units/mL penicillin, and 10% heat‐inactivated newborn calf serum (Invitrogen). Cells were tested for mycoplasma every six months using MycoAlert Detection Kit (Lonza).

### 2.2 IHC (Immunohistochemistry)

The human HNSCC tissue microarrays (paraffin‐embedded), including follow‐up survival information, were provided by SuperBioChips. The arrays underwent incubation with anti‐CUL4B antibody (1:200) in 0.1% Triton X‐100 and 5% bovine serum albumin/PBS (Sigma) for sixteen hours at 4°C. Then, the fixed cells were incubated in 0.1 mol/L Tris‐HCl, pH 7.5, containing 0.05 mol/L acetic acid (chondroitinase reaction buffer) and 0.5 units/mL protease‐free chondroitinase ABC (Sigma) for two hours at 37°C. After three washes, the cells were incubated in blocking solution and stained with 1B5 antibody (1:20) and Alexa 488‐conjugated goat anti‐mouse IgG (1:100, Thermo Fisher Scientific Inc, Waltham, MA, USA). The immunostaining was observed using 3,3‐diaminobenzidine and counterstained with hematoxylin (Sigma) using the UltraVision Quanto Detection System (Thermo Fisher Scientific Inc). The distribution and positive intensity of CUL4B were analyzed by two individuals in a double‐blind experimental design. The staining scores were assigned according to the percentage of positive tumor cells (0, 0%; 1, <25%; 2, 25‐50%; 3, 51‐75%; and 4, >75%) and staining intensity (0, none; 1, weakly stained; 2, moderately stained; and 3, strongly stained).

### 2.3 Quantitative real‐time PCR

Total RNA was isolated using TRIzol reagent (Invitrogen). One microgram of total RNA was used in a reverse transcription reaction using the PrimeScript™ RT Reagent Kit (TaKaRa). Real‐time PCR was performed on the cDNA. The specificity of amplification by the primers was confirmed by sequencing the PCR products. Primers are as followed: CUL4B, forward: 5′‐CCTGGAGTTTGTAGGGTTTGAT‐3′, reverse: 5′‐GAGACGGTGGTAGAAGATTTGG‐3′; β‐actin, forward: 5′‐TTAGTTGCGTTACACCCTTTC‐3′, reverse: 5′‐ACCTTCACCGTTCCAGTTT‐3′.

### 2.4 Transfection

For the overexpression experiments, CUL4B cDNA was subcloned into pcDNA3.1. Cells were transfected with plasmids using Lipofectamine 2000 (Invitrogen). The pcDNA3.1 plasmid was used as a control. Transfected cells were selected with 5 μg/mL G418 for two weeks. For shRNA knockdown experiments, two pLKO/CUL4B‐shRNA plasmids were obtained from Santa Cruz Biotechnology. The short hairpin RNA (shRNA) plasmids were transfected and selected using 3 μg/mL puromycin for two weeks.

### 2.5 Western blotting

Western blotting was performed with antibodies against LOX, MMP2, MMP9 (Cell Signaling Technology), ZO‐1, vimentin, VEGF, β‐actin (Abcam), β‐catenin, cyclin D1, c‐myc, MMP7, and p‐GSK3β Ser9 (Santa Cruz Biotechnology).

### 2.6 Cell proliferation and colony formation

Cells (4 × 10^4^) were seeded into 6‐well plates with culture medium. The analysis of the viable cells was carried out using an MTS assay at 0, 24, 48, and 72 hours. For the anchorage‐dependent colony formation assay, indicated cells were seeded in 6‐well plates and incubated for two weeks. Colonies were fixed with methanol and stained with 0.1% crystal violet (Sigma) and colonies were counted. The colony numbers were counted using Image‐pro 3D Suite software version 5.1.1.38 (Media Cybernetics, Inc, Bethesda, MD, USA).

### 2.7 Cell migration and invasion assay

Transwell inserts for 24‐well plates with porous filters without coating (the pore size was 8 μm) were used for the evaluation of cell migration, and Matrigel (BD Biosciences) porous filters with coating were used for the examination of cell invasion. Briefly, 2 × 10^4 ^cells in serum‐free DMEM (0.2 mL) were seeded into the inserts for 8 hours. And then 0.6 mL DMEM with 10% FBS was added in the lower portion of the chamber as a chemoattractant. The cells that transferred to the lower well of the chamber were stained using crystal violet.

### 2.8 Xenograft models

All animal care and experimental procedures in the current study were approved and guided by Animal Ethics Committee of China Medical University. For the analysis of tumor growth, 5 × 10^6^ JHU‐012 mock transfectants were injected subcutaneously into the left flanks of male C57BL/6 mice, and an equal number of CUL4B transfectants were injected into the right flanks (n = 6). The tumor volumes were observed for 20 days, and the excised tumor tissues were weighed and analyzed by immunohistochemistry. The surgically removed tissues underwent paraffin‐embedding for subsequent experiments.

### 2.9 Statistical analysis

All data analysis was performed using GraphPad Prism VI (San Diego, CA, USA). Student's *t *test was employed. Paired *t *tests were employed to analyze the paired JHU‐012 tumors. The comparisons between CUL4B expression levels and clinicopathological characteristics were made using a two‐sided Fisher's exact test. The log‐rank test and Kaplan‐Meier analysis were employed to analyze overall survival. *P* < 0.05 was considered statistically significant.

## 3 RESULTS

### 3.1 High expression level of CUL4B in HNSCC correlates with poor survival

First, we compared the levels of CUL4B in HNSCC tissues and adjusted normal tissues by quantitative real‐time PCR (qRT‐PCR) and Western blotting. Notably, HNSCC tissues showed significantly higher expression levels of CUL4B in comparison with the adjusted normal tissues (Figure 1A). As CUL4B gene locates in the chromosome X, we analyzed the expression of CUL4B in HNSCC tissues in male and female. Our results showed that CUL4B expression is higher in female HNSCC tissues. However, the statistics is not significant (Figure 1B).

**Figure 1:** Expression of CUL4B in human HNSCC. A, qRT‐PCR analysis of CUL4B mRNA in HNSCC tissues (tumor) and paired normal tissues (normal). B, qRT‐PCR analysis of CUL4B mRNA in male and female HNSCC tissues. C, CUL4B protein level in HNSCC tissues and paired normal tissues were assessed by Western blotting. D, Immunohistochemistry of CUL4B in nontumor and primary HNSCC tissue arrays. Scale bar: 50 μm. E, Kaplan‐Meier analysis of overall survival for patients with HNSCC. The analyses were conducted based on the immunohistochemistry of CUL4B and the survival information provided by the supplier. *P < 0.05

We further randomly chose 5 paired tissue samples to assess CUL4B protein levels by Western blotting. In line with previous studies, we found that the protein levels of CUL4B were increased in the HNSCC tissue samples (Figure 1C). These results were confirmed by immunohistochemistry. CUL4B had a higher expression level in almost every cancer tissue than in nontumor tissues (Figure 1D). To determine whether the expression level of CUL4B was correlated with clinicopathological characteristics, the level of CUL4B expression was classified as either a high expression level (staining index > 6) or a low expression level (staining index ≤ 6). Interestingly, the results revealed that CUL4B was highly expressed in 50% (33/66) of HNSCC tumors, whereas only 11% (1/8) of nontumor tissues expressed high levels of CUL4B. According to the Kaplan‐Meier survival analysis, the survival rate was dramatically lower in HNSCC patients who had high expression levels of CUL4B in comparison with those who had low expression levels of CUL4B (Figure 1E). These data reveal that CUL4B is frequently upregulated in head and neck squamous cell carcinoma and that its expression is associated with high histology grade and poor prognosis.

### 3.2 CUL4B regulates malignant phenotypes and epithelial‐mesenchymal transition in HNSCC cells

To explore the role of CUL4B in malignant phenotypes in HNSCC cells, we analyzed colony formation and cell growth, invasion, and migration. As shown in Figure 2A,B, knockdown of CUL4B significantly inhibited cell growth in JHU‐012 cells, whereas CUL4B overexpression resulted in enhanced growth. Consistently, overexpression of CUL4B increased the number of anchorage‐dependent colonies, whereas knockdown of CUL4B slightly decreased the number of colonies (Figure 2C,D). Interestingly, invasion and migration were dramatically promoted by overexpression of CUL4B, while invasion and migration were decreased by CUL4B knockdown (Figure 2E,H). Cell invasion and morphological changes are tightly associated with epithelial‐mesenchymal transition (EMT). Therefore, we analyzed the levels of epithelial markers, such as ZO‐1 and E‐cadherin, as well as the level of vimentin, which is a mesenchymal marker, using Western blotting. These results strongly suggested that the overexpression of CUL4B suppressed the expression of ZO‐1 and E‐cadherin and increased the expression of vimentin in JHU‐012 cells. In contrast, knockdown of CUL4B increased the expression of E‐cadherin and ZO‐1 but decreased the expression of vimentin in the cells (Figure 2I,J). Together, these data indicate that CUL4B can not only modulate HNSCC cell growth but also regulate colony formation, cell migration and invasion and EMT in vitro.

**Figure 2:** Effects of CUL4B on malignant phenotypes in HNSCC cells. A, Cell viability of JHU‐012 cells transfected with vector or CUL4B was analyzed by MTS assays at different time points. B, Cell viability of sh con or sh CUL4B JHU‐012 cells was analyzed by MTS assays at different time points. C, Effects of CUL4B overexpression on anchorage‐dependent colony formation. Scale bar: 10 mm. D, Effects of CUL4B knockdown on anchorage‐dependent colony formation. Scale bar: 10 mm. E, CUL4B overexpression regulated transwell cell invasion and F, Matrigel invasion. Scale bar: 50 μm. G, CUL4B knockdown regulated transwell cell invasion and H, Matrigel invasion. Scale bar: 50 μm. I, Expression of epithelial markers, E‐cadherin and ZO‐1, and mesenchymal markers, vimentin, was analyzed by Western blotting in vector or CUL4B‐transfected JHU‐012 cells. J, Expression of epithelial markers, E‐cadherin and ZO‐1, and mesenchymal markers, vimentin, was analyzed by Western blotting in sh con or sh CUL4B JHU‐012 cells. *P < 0.05; **P < 0.01

### 3.3 CUL4B enhances the activation of the Wnt/β‐catenin signaling pathway

Next, we found that the knockdown of CUL4B in JHU‐012 cells obviously decreased the protein and mRNA levels of β‐catenin, cyclin D1, c‐myc, and MMP7. Overexpression of CUL4B increased the protein and mRNA levels of MMP7, c‐myc, cyclin D1, and β‐catenin (Figure 3A‐C). These results support the idea that CUL4B regulates the Wnt/β‐catenin signaling pathway. To reinforce the evidence of this regulation, the level of the active form of β‐catenin was examined. The level of activated β‐catenin (nonphospho β‐catenin (Ser33/37/Thr41)) was significantly increased in cells overexpressing CUL4B and reduced in JHU‐012 cells lacking CUL4B (Figure 3D). The effect of CUL4B on the activity of β‐catenin signaling was also analyzed using the TOP/FOP Flash assay, which is a well‐established dual‐luciferase reporter assay for TCF/β‐catenin. The TOP Flash reporter contains TCF‐responsive sites. However, the FOP Flash reporter contains mutant TCF binding sites, which serve as negative controls. Based on the results, we found that TOP Flash luciferase activity was significantly reduced when CUL4B was knocked down, while the overexpression of CUL4B promoted the activation of the TCF reporter (Figure 3E,F). Therefore, the above findings indicate that CUL4B plays a key role as a positive mediator of Wnt/β‐catenin activity.

**Figure 3:** CUL4B enhances Wnt/β‐catenin signaling in HNSCC cells. A, mRNA level of β‐catenin, cyclin D1, c‐myc, and MMP7 in vector or CUL4B overexpressed JHU‐012 cells was determined by qRT‐PCR. B, mRNA level of β‐catenin, cyclin D1, c‐myc, and MMP7 in sh con or sh CUL4B JHU‐012 cells was determined by qRT‐PCR. C, Protein level of β‐catenin, cyclin D1, c‐myc, and MMP7 in the indicated group was determined by qRT‐PCR and Western blotting. (D) Levels of the active form of β‐catenin in JHU‐012 cells with knockdown or overexpression of CUL4B. E and F, The activity of TCF/β‐catenin reporter (TOP/FOP Flash) in CUL4B‐knockdown (E) and CUL4B‐overexpressing cells (F). *P < 0.05; **P < 0.01

### 3.4 Wnt/β‐catenin signaling regulates CUL4B function in HNSCC cells

We then treated HNSCC cells that were overexpressing CUL4B with XAV‐939, a Wnt/β‐catenin signaling inhibitor. We found that cell growth was significantly suppressed following XAV‐939 treatment in cells overexpressing CUL4B (Figure 4A). Furthermore, the results from transwell assays showed that blockade of the Wnt/β‐catenin pathway significantly abolished CUL4B‐enhanced cell migration and invasion (Figure 4B,C).

**Figure 4:** Wnt/β‐catenin signaling regulates CUL4B functions in HNSCC cells Effects of XAV‐939, on CUL4B‐enhanced cell proliferation (A), migration (B), and invasion (C). Scale bar: 50 μm. Cells were treated with XAV‐939 or DMSO during the migration and invasion assays. **P < 0.01

### 3.5 CUL4B promotes tumor growth in xenograft model

To investigate the effects of CUL4B on tumor growth in vivo, we established xenograft tumors with CUL4B‐, vector‐, sh‐CUL4B‐, and shRNA‐con‐transfected cells in BALB/c nude mice. Compared with that of the shRNA‐con group, the tumor volume of the sh‐CUL4B group was significantly smaller at the 20th day after inoculation. Similarly, compared with the control group, the CUL4B group had greater growth. The shRNA‐con group and control group tumors were not significantly different in growth (Figure 5A,B). Compared to the shRNA‐con group, the sh‐CUL4B group had lower tumor weights. The tumor weight was higher in the CUL4B group than in the control group. In addition, no difference in tumor weight was observed between the shRNA‐con and control groups (Figure 5C,D). CUL4B expression was confirmed by Western blotting (Figure 5E,F). In addition, β‐catenin was found upregulated in the CUL4B group compared to the control group (Figure 5E). Moreover, compared with the shRNA‐con group, CUL4B reduced in the sh‐CUL4B group (Figure 5F). Immunohistochemistry analysis revealed that the knockdown of CUL4B obviously reduced tumor growth, as revealed by Ki67 staining, while CUL4B overexpression promoted tumor growth (Figure 5G,H). Furthermore, the expression of MMP7, c‐myc, cyclin D1, and β‐catenin was upregulated in CUL4B‐overexpressing group in comparison with the control group (Figure 5I).

**Figure 5:** CUL4B enhanced tumor growth in vivo. A, Tumor volume in sh con and sh CUL4B tumors. B, Tumor volume in sh con and sh CUL4B tumors. C, Tumor weight in vector and CUL4B tumors. D, Tumor weight in sh con and sh CUL4B tumors. E, CUL4B and β‐catenin expression in vector and CUL4B tumor was analyzed by Western blotting. F, CUL4B and β‐catenin expression in sh con and sh CUL4B tumor was analyzed by Western blotting. G, Expression of Ki‐67 (cell proliferation marker) in vector and CUL4B tumors was analyzed by immunohistochemistry. Scale bar: 50 μm. *P < 0.05. H, Expression of Ki‐67 in sh con and sh CUL4B tumors was analyzed by immunohistochemistry. Scale bar: 50 μm. *P < 0.05. I, Expression of MMP7, c‐myc, cyclin D1, and β‐catenin in vector and CUL4B tumors was analyzed by immunohistochemistry. Scale bar: 50 μm. *P < 0.05.

### 3.6 Angiogenesis is enhanced by high expression levels of CUL4B in HNSCC tissues

The α‐SMA‐ and CD31‐staining results demonstrated that there were pericytes and vascular endothelial cells in the blood vessels. There were more α‐SMA‐ and CD31‐positive cells in tumors overexpressing CUL4B in comparison with the control tumors (Figure 6A), suggesting that high expression levels of CUL4B facilitate tumor angiogenesis. We next investigated the levels of proteins that were related to tumor metastasis and angiogenesis in the sera of mice bearing control and CUL4B overexpressing tumors. Notably, the protein levels of LOX, MMP9, and VEGF in the sera of mice bearing tumors overexpressing CUL4B were increased compared to those of control mice (Figure 6B). Additionally, the levels of LOX, VEGF, and MMP9 were markedly elevated in tumors overexpressing CUL4B compared to control tumors (Figure 6C), demonstrating that the elevated levels of those proteins in the serum were probably caused by the enhanced expression of CUL4B in tumors. These results strongly suggest that metastasis and angiogenesis are stimulated by high expression levels of CUL4B in HNSCC via increased expression of MMP9, LOX, and VEGF.

**Figure 6:** CUL4B overexpression promotes angiogenesis. A, Immunofluorescent staining of CD31 (red) and α‐SMA (red) merged with nuclei (blue) in JHU‐012‐Ctrl and JHU‐012‐CUL4B tumors. Scale bar: 50 μm. B, VEGF, MMP9, and LOX in sera from JHU‐012‐CUL4B tumor‐bearing mice and JHU‐012‐Ctrl mice were analyzed by Western blotting. C, The expression of MMP9, VEGF, and LOX in JHU‐012‐CUL4B and JHU‐012‐Ctrl tumors as assessed by immunohistochemistry. Scale bar: 50 μm

## 4 DISCUSSION

CRL4B is a component of CRL4B that can target different substrates for protein modification or proteasomal degradation.^13^ Recently, high expression levels of CUL4B have been found in a variety of human malignancies, such as cervical cancer, esophageal cancer, liver cancer, and osteosarcoma, and these enhanced expression levels are positively correlated with tumor progression.^11^, ^14^, ^15^, ^16^ Our study showed that CUL4B upregulation in HNSCC tissues was associated with worse tumor grade and shorter survival. EMT is considered a key step in tumor invasion and metastasis. HNSCC, which is known to have EMT characteristics, shows more vascular invasion and metastases, as well as a poorer prognosis.^17^, ^18^ It has been reported that CUL4B knockdown in NSCLC inhibits EMT progression and decreases the level of c‐myc, cyclin D1, and β‐catenin.^19^ In addition, CUL4B overexpression significantly enhanced the growth of hepatocytes in liver cells in a recently established mouse model.^20^ Here, we investigated whether CUL4B expression regulates EMT in HNSCC cells to determine whether CUL4B drives tumor proliferation.

Recent reports have suggested the abnormal activation of Wnt/β‐catenin signaling in several human malignancies including HNSCC.^21^, ^22^ Abnormal activation of the Wnt/β‐catenin signaling pathway has been shown to be closely related to the oncogenic effects of various types of cancers.^23^, ^24^ Wnt/β‐catenin signaling activity is associated with poor histological differentiation, aggressive invasion, and chemoresistance in HNSCC.^25^ Moreover, targeting Wnt/β‐catenin signaling is an attractive option for the treatment of various types of human cancers such as HNSCC.^22^, ^26^ Previous studies have shown that CUL4B functions as a positive regulator of Wnt/β‐catenin signaling by transcriptionally reducing several Wnt antagonists including DKK1 and PPP2R2B, leading to protect of β‐catenin from GSK‐3‐mediated degradation.^11^ In the present study, CUL4B activated the Wnt/β‐catenin pathway, and CUL4B‐induced cell migration, invasion, and metastasis were inhibited by Wnt/β‐catenin inhibitors. CUL4B knockdown significantly decreased the level of β‐catenin and the level of the target gene, whereas overexpression of CUL4B increased the accumulation of β‐catenin and the level of target gene. These findings provide new information regarding the function of CUL4B in HNSCC; it also provides clues for the development of novel therapies for HNSCC. Although we could not exclude the effects of other growth factors or proteinases from our experimental conditions, CUL4B‐mediated tumor malignancy may mainly occur through the activation of the Wnt/β‐catenin pathway. Therefore, it is necessary to understand in more detail the functions and regulatory mechanisms involved in the activation of the Wnt/β‐catenin signaling pathway in HNSCC in order to improve the efficacy of targeted therapies. Therefore, targeting CUL4B in a tumor microenvironment may produce similar results as targeting multiple kinases in cancer cells. Taken together, our results suggest that CUL4B regulates Wnt/β‐catenin signaling, which is involved in the malignant behavior of CUL4B‐induced HNSCC cells.

## CONFLICT OF INTEREST

The authors have declared that no conflicts of interest exist.

## References

[1] Safdari Y , Khalili M , Farajnia S , Asgharzadeh M , Yazdani Y , Sadeghi M . Recent advances in head and neck squamous cell carcinoma–a review. Clin Biochem. 2014;47(13‐14):1195‐1202.2491205010.1016/j.clinbiochem.2014.05.066

[2] Sano D , Oridate N . The molecular mechanism of human papillomavirus‐induced carcinogenesis in head and neck squamous cell carcinoma. Int J Clin Oncol. 2016;21(5):819‐826.2733927010.1007/s10147-016-1005-x

[3] Price KA , Cohen EE . Current treatment options for metastatic head and neck cancer. Curr Treat Options Oncol. 2012;13(1):35‐46.2225288410.1007/s11864-011-0176-y

[4] Sacco AG , Cohen EE . Current treatment options for recurrent or metastatic head and neck squamous cell carcinoma. J Clin Oncol. 2015;33(29):3305‐3313.2635134110.1200/JCO.2015.62.0963

[5] Chawla S , Kim S , Loevner LA , et al. Prediction of disease‐free survival in patients with squamous cell carcinomas of the head and neck using dynamic contrast‐enhanced MR imaging. AJNR Am J Neuroradiol. 2011;32(4):778‐784.2134996910.3174/ajnr.A2376PMC7965863

[6] Dahiya K , Dhankhar R . Updated overview of current biomarkers in head and neck carcinoma. World J Methodol. 2016;6(1):77‐86.2701832410.5662/wjm.v6.i1.77PMC4804254

[7] Sepiashvili L , Hui A , Ignatchenko V , et al. Potentially novel candidate biomarkers for head and neck squamous cell carcinoma identified using an integrated cell line‐based discovery strategy. Mol Cell Proteomics. 2012;11(11):1404‐1415.2291822610.1074/mcp.M112.020933PMC3494179

[8] Hannah J , Zhou P . Distinct and overlapping functions of the cullin E3 ligase scaffolding proteins CUL4A and CUL4B. Gene. 2015;573(1):33‐45.2634470910.1016/j.gene.2015.08.064PMC5110433

[9] Kerzendorfer C , Hart L , Colnaghi R , et al. CUL4B‐deficiency in humans: understanding the clinical consequences of impaired Cullin 4‐RING E3 ubiquitin ligase function. Mech Ageing Dev. 2011;132(8–9):366‐373.2135284510.1016/j.mad.2011.02.003

[10] Mok MT , Cheng AS . CUL4B: a novel epigenetic driver in Wnt/beta‐catenin‐dependent hepatocarcinogenesis. J Pathol. 2015;236(1):1‐4.2566453310.1002/path.4512

[11] Yuan J , Han B , Hu H , et al. CUL4B activates Wnt/beta‐catenin signalling in hepatocellular carcinoma by repressing Wnt antagonists. J Pathol. 2015;235(5):784‐795.2543088810.1002/path.4492

[12] Mao XW , Xiao JQ , Xu G , et al. CUL4B promotes bladder cancer metastasis and induces epithelial‐to‐mesenchymal transition by activating the Wnt/beta‐catenin signaling pathway. Oncotarget. 2017;8(44):77241‐77253.2910038410.18632/oncotarget.20455PMC5652777

[13] Lee J , Zhou P . Pathogenic role of the CRL4 ubiquitin ligase in human disease. Front Oncol. 2012;2:21.2264978010.3389/fonc.2012.00021PMC3355902

[14] Yang Y , Liu R , Qiu R , et al. CRL4B promotes tumorigenesis by coordinating with SUV39H1/HP1/DNMT3A in DNA methylation‐based epigenetic silencing. Oncogene. 2015;34(1):104‐118.2429268410.1038/onc.2013.522

[15] Hu H , Yang Y , Ji Q , et al. CRL4B catalyzes H2AK119 monoubiquitination and coordinates with PRC2 to promote tumorigenesis. Cancer Cell. 2012;22(6):781‐795.2323801410.1016/j.ccr.2012.10.024

[16] Chen Z , Shen BL , Fu QG , et al. CUL4B promotes proliferation and inhibits apoptosis of human osteosarcoma cells. Oncol Rep. 2014;32(5):2047‐2053.2518918610.3892/or.2014.3465

[17] Smith A , Teknos TN , Pan Q . Epithelial to mesenchymal transition in head and neck squamous cell carcinoma. Oral Oncol. 2013;49(4):287‐292.2318239810.1016/j.oraloncology.2012.10.009PMC3586749

[18] Chen C , Zimmermann M , Tinhofer I , Kaufmann AM , Albers AE . Epithelial‐to‐mesenchymal transition and cancer stem(‐like) cells in head and neck squamous cell carcinoma. Cancer Lett. 2013;338(1):47‐56.2277153510.1016/j.canlet.2012.06.013

[19] Wang X , Chen Z . Knockdown of CUL4B suppresses the proliferation and invasion in non‐small cell lung cancer cells. Oncol Res. 2016;24(4):271‐277.2765683810.3727/096504016X14666990347473PMC7838745

[20] Yuan J , Jiang B , Zhang A , et al. Accelerated hepatocellular carcinoma development in CUL4B transgenic mice. Oncotarget. 2015;6(17):15209‐15221.2594583810.18632/oncotarget.3829PMC4558146

[21] Lee SH , Koo BS , Kim JM , et al. Wnt/beta‐catenin signalling maintains self‐renewal and tumourigenicity of head and neck squamous cell carcinoma stem‐like cells by activating Oct4. J Pathol. 2014;234(1):99‐107.2487103310.1002/path.4383

[22] Padhi S , Saha A , Kar M , et al. Clinico‐pathological correlation of beta‐catenin and telomere dysfunction in head and neck squamous cell carcinoma patients. J Cancer. 2015;6(2):192‐202.2565372110.7150/jca.9558PMC4314668

[23] Liang Y , Feng Y , Zong M , et al. Beta‐catenin deficiency in hepatocytes aggravates hepatocarcinogenesis driven by oncogenic beta‐catenin and MET. Hepatology. 2017;67(5):1807‐1822.10.1002/hep.29661PMC590614729152756

[24] Li P , Liu W , Xu Q , Wang C . Clinical significance and biological role of Wnt10a in ovarian cancer. Oncol Lett. 2017;14(6):6611‐6617.2916369210.3892/ol.2017.7062PMC5686444

[25] Schultz JD , Sommer JU , Hoedt S , et al. Chemotherapeutic alteration of beta‐catenin and c‐kit expression by imatinib in p16‐positive squamous cell carcinoma compared to HPV‐negative HNSCC cells in vitro. Oncol Rep. 2012;27(1):270‐280.2199376610.3892/or.2011.1499

[26] Böhrnsen F , Fricke M , Sander C , Leha A , Schliephake H , Kramer FJ . Interactions of human MSC with head and neck squamous cell carcinoma cell line PCI‐13 reduce markers of epithelia‐mesenchymal transition. Clin Oral Invest. 2015;19(5):1121‐1128.10.1007/s00784-014-1338-725346374

